This article has been retracted.

# Impact of different mulching treatments on weed flora and productivity of maize (*Zea mays* L.) and sunflower (*Helianthus annuus* L.)

**DOI:** 10.1371/journal.pone.0266756

**Published:** 2022-04-15

**Authors:** Mubshar Hussain, Syed Nasir Abbas Shah, Muhammad Naeem, Shahid Farooq, Khawar Jabran, Saleh Alfarraj

**Affiliations:** 1 Department of Agronomy, Bahauddin Zakariya University, Multan, Pakistan; 2 School of Veterinary and Life Sciences, Murdoch University, Murdoch, WA, Australia; 3 The Urban Unit, Shaheen Complex, Garhi Shahu, Lahore, Punjab, Pakistan; 4 Faculty of Agriculture, Department of Plant Protection, Harran University, Şanlıurfa, Turkey; 5 Department of Plant Production and Technologies, Niğde Ömer Halisdemir University, Niğde, Turkey; 6 Zoology Department, College of Science, King Saud University, Riyadh, Saudi Arabia; Mendel University of Agriculture and Forestry: Mendelova univerzita v Brne, CZECH REPUBLIC

## Abstract

The concerns on weed control through herbicides are increasing due to their negative impacts on environment and human health. Therefore, alternative weed management methods are inevitable for sustainable crop production and lowering the negative consequences of herbicides. Mulching is an environment-friendly weed management approach capable of substituting herbicides to significant extent. Therefore, this study evaluated the role of different mulching treatments on suppressing weed flora in maize (*Zea mays* L.) and sunflower (*Helianthus annuus* L.) crops. Furthermore, the impact of different mulching treatments on the productivity of both crops was also investigated. Three mulch treatments, i.e., plastic mulch (PLM), sorghum mulch (SM) and paper mulch (PM) along with two controls, i.e., weed-free (WF) and weedy-check (WC) were included in the study. Different mulch treatments significantly altered weed flora in both crops. The PLM and PM resulted in the highest suppression (43–47%) of weed flora compared to WC treatment in both crops. The highest and the lowest weed diversity was recorded for WC and WF treatments, respectively. Different allometric traits, i.e., leaf area index, crop growth rate and root length of both crops were significantly improved by PLM as compared to the WC. Overall, maize crop recorded higher density of individual and total weeds compared to sunflower with WC treatment. The density of individual and total weeds was significantly lowered by PLM compared to WC treatment in both crops. Similarly, higher growth and yield-related traits of both crops were noted with PLM compared to the rest of the mulching treatments. Results of the current study warrant that PLM could suppress weed flora and improve the productivity of both crops. However, PLM alone could not provide 100% control over weed flora; therefore, it should be combined with other weed management approaches for successful weed control in both crops.

## Introduction

Maize (*Zea mays* L.) is globally ranked 3^rd^ among cereal crops in terms of area under cultivation. It is primarily cultivated for grain and forage purposes around the world [1,2]. Grain maize cultivated on an area of 1.41 million hectares in Pakistan during 2020 with total grains production of 8.46 million tones, which contributed 0.5% towards country’s gross domestic product [3]. Maize is also called ‘queen of cereals’ due to its wider adaptability to diverse climatic conditions and higher production [4]. The grains of maize crop are highly nutritious and contain significant amounts of carbohydrates (44.60–69.60%), protein (9.87%), minerals (1.10–2.95%), fat (2.17–4.43%) and fiber (2.10–26.70%) [5]. Sunflower (*Helianthus annuus* L.) is 4^th^ most important oilseed crop globally in terms of area under cultivation and its seeds contain high oil and protein contents [6]. Sunflower seeds contain 28–32% protein and 36–52% oil contents [7]. The total edible oil production in Pakistan was 0.50 million tons during 2018–19, while 2.42 million tons of oil costing 192.20 billion rupees was imported to fulfill the domestic edible oil requirements of the country [3].

Crop productivity is significantly influenced by several biotic and abiotic factors [8–10]. Weeds are among the major constraints in crop production, which significantly reduce yield and quality of the produce [11–13]. Weeds compete with crop plants for nutrients, water, light and space, which ultimately result in reduced crop yield [14–17]. Weed infestation also exerts negative impacts on economy and causes environmental and health issues in terrestrial ecosystems [18]. Maize crop (like all crops) had a specific critical period during which weed control is necessary to reduce yield losses [19,20]. Weeds can be controlled by depleting soil seed bank through integrated weed management methods comprising of herbicides, mulching, tillage operations, sowing methods, and hand weeding [21].

Mulching is an important technology widely used in orchards and agricultural system to conserve soil moisture and improve weed control in row crops [22,23]. Furthermore, mulching is also aimed at reducing soil erosion [24]. Different mulch materials, i.e., organic (e.g. straw or wood chips), polyethylene foils, polypropylene nonwoven fabrics, gravels, biodegradable plastic foils are used to serve these purposes [25,26]. Plastic mulching plays an important role in crop growth and development as it conserves soil moisture and decreases weed infestation [27–29]. Furthermore, plastic mulching adjusts soil temperature, improves crop yield, and decreases costs incurred on herbicides and fertilizers [30]. Similarly, paper mulching conserves soil moisture through reduced water evaporation. Furthermore, it improves soil quality when returned to field after harvesting in the following season [31].

Weeds can be managed by exploiting allelopathic potential of crops using mulches [32], residues’ incorporation [33], intercropping [34], crop rotation [13,15,16], cover crops and allelopathic crop water extracts [35,36]. Different types of phenolics, i.e., protocatechuic acid, syringic acid, chlorogenic acid, p-hydroxybenzoic acid, vanillic acid, ferulic acid, p-coumaric acid, gallic acid, caffeic acid and benzoic acid have been recognized from sorghum crop [37]. Owing to existence of these phenolics, sorghum water extracts and sorghum mulch may help in decreasing weed infestation [13,38]. Therefore, using mulches of allelopathic crops could provide significant control over weed flora. However, mulch materials obtained from allelopathic crops like sorghum has not been tested on large scale.

Weed management in sunflower and maize is highly reliant on herbicides, although several cultural and mechanical methods are also used. Mulching has been used in different countries to suppress weed flora in both crops. For example, Latify et al. [39] intercropped *Fagopyrum esculentum*, *Medicago scutellate* and *Vicia villosa* as living mulch in different cultivars of sunflower to suppress weed flora. The cultivars and living mulches significantly differed in their ability to decrease weed infestation. The lowest level of weed infestation was noted for *V*. *villosa* living mulch in Azargol cultivar. Similarly, Latify et al. [40], suggested that weed suppression ability of different cultivars significantly differ; therefore, proper cultivar and mulch combination is necessary for efsfective weed management. Uwah et al. [41], reported that use of organic mulch (6 or 8 tons/ha) suppressed weed flora and improved grain yield of maize crop. However, plastic and paper mulch have been rarely tested for suppressing weed flora in maize and sunflower.

Mulching is an important technique to suppress weed flora and improve crop yield. However, the role of different mulches in suppressing weed flora and improving the productivity of maize and sunflower crops has rarely been tested. Therefore, this field study was conducted to evaluate the role of different mulch materials in improving yield of maize and sunflower, and suppressing weed flora present in these crops. It was hypothesized that mulch materials will significantly differ from each other in their ability to suppress weed flora and improve crop productivity. It was further hypothesized that sorghum mulch will provide better weed control compared to plastic and paper mulches. The results of the study will help to improve weed control in maize and sunflower crops. Furthermore, the results will help to reduce the herbicide use and associated negative impacts on environment and human health.

## Materials and methods

### Experimental site and soil

This field study was carried out at Agronomic Research Farm, Bahauddin Zakariya University (BZU), Multan Pakistan (71.43° E, 30.2° N and 122 m above sea level.) during maize and sunflower growing seasons of 2018. Experimental soil was clay-loam with 7.9 pH, 2.32 mS cm^-1^ ECe, 0.65% organic matter content, 0.03% total nitrogen, 7.30 ppm available phosphorus and 218 ppm available potassium. The weather data of the experimental field during the study period are given in Fig 1.

**Fig 1:** Weather data of the experimental site during maize and sunflower growth seasons.

### Experimental details

Three different mulch materials, i.e., plastic mulch (PLM), sorghum mulch (SM) and paper mulch (PM), and two controls, i.e., weed-free (WF) and weedy-check (WC) were tested for their ability to suppress weed flora and improve the productivity of maize and sunflower. Weeds were totally removed throughout growth period of both crops in WF treatment, while allowed to grow for the entire cropping periods in WC treatment. Black plastic mulch and packing paper were placed between crop rows in PLM and PM treatments, respectively. In SM treatment, sorghum plants were chopped (5 tones ha^-1^), dried and placed between the rows of both crops. Thin soil layer was also placed or mixed in these mulches to avoid the movement due to wind or water. The experiment had three replications and laid out according to randomized complete block design (RCBD). The net plot size was 5.0 m × 3.0 m.

### Crop husbandry

Initially, pre-soaking irrigation of 10 cm was applied to the experimental field. When soil achieved feasible moisture level, seedbeds for each crop were prepared by cultivating the field two times followed by planking. Maize (cultivar ‘P1429’) and sunflower (Hybrid cultivar ‘NK-SINGI’) were sown on February 22, 2018, by using hand drill in 75 cm apart rows using seed rate of 6 and 20 kg/ha for sunflower and maize, respectively. Irrigation was done according to the necessity of crops to avoid moisture stress. The NPK fertilizer was applied at the rate of 150-100-60 kg/ha in sunflower and 100-60-40 kg/ha in maize by using urea, diammonium phosphate (DAP), sulphate of potash (SOP) as source, for N, P and K, respectively. Furadan (20 kg/ha) was used at 4–5 leaf stage in maize to save the crop from the attack of stem borer. Sucking and chewing insects were controlled by spraying Match (Leofenoran 50 g/L, 500 ml/ha) and Bifenthren (650 ml ha^-1^). Both crops were harvested at their harvest maturity.

### Observations

Data related to density of individual weeds and weed diversity were noted from each experimental unit at 35, 55 and 75 DAS (days after sowing). Data on weed density were recorded from three randomly selected locations in each experimental unit by using 1 m^2^ quadrate. Overall (total) weed density was computed by adding the densities of all individual weeds. Likewise, densities of broadleaved and grassy weeds were recorded by adding their individual densities. Six weed species were identified throughout the study. The identified weed species were *Trianthima portulacastrum* L., *Cyperus rotundus* L., *Chenopodium album* L., *Parthinum hysterophorus* L., *Remux dentatus* L. and *Cyndon dactylon* L.

Randomly selected two plants from each experimental unit were harvested after every twenty days to estimate leaf area index (LAI) and crop growth rate (CGR). The sampling was started at 35 DAS and terminated at 95 DAS. The leaves of harvested plants were detached, and their fresh weights were recorded. Afterwards, leaf area per plant was noted with leaf area meter (DT Area Meter, model MK2) and converted to total leaf area of the harvested samples by unitary method. The LAI was determined by following Watson [42]. Furthermore, harvested samples were chaffed, sundried for 3 days and oven-died at 75°C for 72 hours. Afterwards, CGR was determined by following Hunt [43]. Dry biomass produced by the harvested plants at each harvest was used to compute CGR.

Two randomly selected plants (of both crops) were uprooted carefully, and their root lengths were measured by using measuring tape at 35, 55 and 75 DAS. Three plants were randomly selected, and their heights were measured. Cob length, number of rows and grains per cob were recorded from five randomly selected cobs. Three random samples of 1000-grains were taken from each plot and weighed on an electric balance. The plants in each plot were harvested, tied into bundles and their weight was recoded with spring balance to measure biological yield. Afterwards, all cobs were detached from the plants and sundried for 3 days. Cobs were threshed manually, and weight of the resulting grains was recorded for obtaining grain yield. Biological and grain yields were converted into tons ha^-1^ by using unitary method. Harvest index was calculated as the ratio of grain yield to the biological yield expressed in percentage. Head diameter and number of achenes per head of sunflower were determined from three randomly selected plants and averaged.

### Statistical analysis

The collected data were statistically analyzed by Fisher’s analysis of variance (ANOVA) technique [44]. Two-way ANOVA was used to test the significance in weeds-related data. However, one way ANOVA was used to infer the differences among growth and yield-related traits of both crops due to different nature. Least significant difference (LSD) post-hoc test was used to compare the treatments’ means where ANOVA indicated significant differences. All statistical computations were done on SPSS statistical software [45]. The WF treatment was excluded while analyzing the weed-related data since no weeds were recorded. The minimal dataset used to report the results have been given in S1 Table.

## Results

### Weeds diversity (m^-2^)

Different mulch treatments significantly altered weeds’ diversity in both crops (Fig 2). Overall, WF and WC treatments (controls) resulted in the lowest and the highest weed diversity in both crops. However, among mulching treatments, the highest weed diversity was recorded for SM, while PLM resulted in the lowest weed diversity in both crops at 35, 55 and 75 DAS (Fig 2).

**Fig 2:** Impact of different mulching treatments on weed diversity in maize and sunflower at 35, 55 and 75 DAS. In the legend, WC = Weedy check (control), WF = Weed free (control), Pl-M = Plastic mulch, SM = Sorghum mulch, PM = Paper mulch.

### Density of total, broadleaved and grassy weed species (m^-2^)

Different mulching treatments had significant effect on the density of total, broadleaved and grassy weed species (Table 1). The highest total weeds density was recorded for WC treatment in maize crop, while PLM and PM treatments in sunflower resulted in the lowest density at 35, 55 and 75 DAS (Table 1). The highest density of broadleaved weed species was noted for WC treatment in maize crop at all sampling dates, whereas PLM and PM resulted in the lowest density of broadleaved weed species in sunflower crop (Table 1). Likewise, the highest density of grassy weed species was recorded in maize crop with WC treatment, while the lowest were noted in sunflower crop with PLM, SM and PM at 35 and 75 DAS. However, maize crop with WC treatment recorded the highest density of grassy weed species at 55 DAS, while maize crop with PM and sunflower crop with PLM recorded the lowest density (Table 1).

**Table 1:** Impact of different mulching treatments on the density (m^-2^) of total, broadleaved and grassy weed spices in maize and sunflower at 35, 55 and 75 DAS.

Treatments	35 DAS		55 DAS		75 DAS	
	Maize	Sunflower	Maize	Sunflower	Maize	Sunflower
	Total weeds					
**Weedy-check**	93.66 a	51.33 c	102.33 a	57.66 c	108.67 a	63.66 c
**Plastic mulch**	51.66 c	29.00 e	54.00 c	33.30 f	57.66 cd	36.00 f
**Sorghum mulch**	67.66 b	39.33 d	72.66 b	45.0 d	74.00 b	48.00 e
**Paper mulch**	49.66 c	34 de	43.33 de	36.66 ef	56.66 d	40.00 f
**LSD at p≤0.05**	5.92		8.20		5.52	
	**Broadleaved weeds**					
**Weedy-check**	59.00 a	25.00 de	68.33 a	30.33 cd	69.66 a	32.00 c
**Plastic mulch**	31.33 c	13.33 g	33.33 c	16.66 e	35.66 c	18.66 e
**Sorghum mulch**	42.33 b	21.00 ef	46.66 b	25.00 d	46.33 b	26.00 d
**Paper mulch**	28.66 cd	16.66 fg	30.66 cd	18.66 e	32.66 c	20.33 e
**LSD at p≤0.05**	5.13		5.82		5.57	
	**Grassy weeds**					
**Weedy-check**	34.66 a	26.33 b	34.00 a	27.33 ab	39.00 a	31.66 b
**Plastic mulch**	20.33 bc	15.66 c	20.66 b	16.33 d	22.00 de	17.33 e
**Sorghum mulch**	25.33 b	18.33 c	26.00 b	20.00 bcd	27.66 bc	22.00 de
**Paper mulch**	21.00 bc	17.33 c	12.66 d	18.00 cd	24.00 cd	19.66 de
**LSD at p≤0.05**	6.09		7.42		5.52	

Means not having common letter for individual and interactive effects significantly vary from each other at p≤0.05.

### Density of individual weed species

Various mulch treatments exerted significant effect on density of individual weed species recorded in both crops (Table 2). The PLM significantly reduced the density of *Trianthima portulacastrum* L. compared to the rest of the mulching treatments. In case of *Cyperus rotundus* L., PLM recorded the lowest density at 35 and 75 DAS, which was statistically similar with SM and PM in sunflower crop. However, the lowest density of this weed was noted for PM in maize crop which was statistically similar to PLM and SM in sunflower crop at 55 DAS. Different mulch treatments and crops had non-significant effect on the densities of *Parthinum hysterophorus* L., *Remux dentatus* L., *Cynodon dactylon* L., and *Chenopodium album* L.; however, PLM treatment performed better as compared to other mulch treatments at all data sampling dates (Table 2).

**Table 2:** Impact of different mulching treatments on the density (m^-2^) of individual weed species in maize and sunflower at 35, 55 and 75 DAS.

Treatments	35 DAS		55 DAS		75 DAS	
	Maize	Sunflower	Maize	Sunflower	Maize	Sunflower
	*Cynodon dactylon* L.					
**Weedy-check**	3.33 a	4.00 a	1.33 ab	1.66 a	1.66 a	1.33 ab
**Plastic mulch**	0.66 b	1.00 b	0.33 bc	-	-	-
**Sorghum mulch**	1.00 b	1.33 b	0.33 bc	1.00 abc	0.33 c	0.66 bc
**Paper mulch**	-	1.33 B	-	1.00 abc	0.66 bc	0.33 c
**LSD at p≤0.05**	1.93		1.17		0.72	
	***Remux dentatus* L.**					
**Weedy-check**	1.33 a	1.00 ab	1.33 a	1.00 ab	1.00 a	1.00 a
**Sorghum mulch**	0.33 bc	-	-	-	0.33 bc	-
**Paper mulch**	0.66 abc	0.66 abc	0.66 bc	0.66 bc	0.33 bc	0.66 ab
**Weedy-check**	0.33 bc	0.33 bc	0.33 ab	0.33 ab	-	-
**LSD at p≤0.05**	0.91		1.07		0.57	
	***Parthinum hysterophorus* L.**					
**Weedy-check**	1.33 a	1.00 ab	1.67 a	0.66 b	1.00 a	0.66 ab
**Sorghum mulch**	0.33 ab	-	0.33 b	-	-	-
**Paper mulch**	0.66 ab	0.33 ab	0.66 b	0.33 b	0.33 bc	0.33 bc
**Weedy-check**	0.66 ab	0.33 ab	0.33 b	-	0.66 ab	-
**LSD at p≤0.05**	1.10		0.93		0.63	
	***Chenopodium album* L.**					
**Weedy-check**	1.66 a	1.00 ab	1.66 a	1.33 ab	1.66 a	1.00 ab
**Sorghum mulch**	0.34 b	0.33 b	0.33 bc	0.33 bc	-	-
**Paper mulch**	0.66 ab	0.66 ab	1.00 abc	0.66 abc	1.00 abc	0.66 bc
**Weedy-check**	0.66 ab	0.33 b	0.66 abc	0.33 bc	0.66 bc	-
**LSD at p≤0.05**	1.23		1.09		0.92	
	***Cyperus rotundus* L.**					
**Weedy-check**	31.33 a	22.33 b	32.66 a	25.66 ab	37.33 a	30.33 b
**Sorghum mulch**	19.66 bcd	14.66 e	20.33 bc	16.33 cd	22.00 cde	17.33 e
**Paper mulch**	24.33 b	17.00 cde	25.66 ab	19.00 bcd	27.33 bc	21.33 de
**Weedy-check**	21.00 bc	16.00 de	12.66 d	17.00 cd	23.33 cd	19.33 de
**LSD at p≤0.05**	4.92		7.20		5.50	
	***Trianthima portulacastrum* L.**					
**Weedy-check**	55.33 a	23.00 d	63.66 a	27.33 de	66.00 a	29.33 de
**Sorghum mulch**	30.66 c	13.00 f	32.66 c	16.33 f	35.33 c	18.66 g
**Paper mulch**	40.66 b	18.33 e	44.33 b	23.33 e	44.66 b	24.33 ef
**Weedy-check**	27.00 cd	15.66 ef	29.33 cd	18.00 f	31.33 cd	20.33 fg
**LSD at p≤0.05**	4.43		5.20		5.40	

Means not having common letter for individual and interactive effects significantly vary from each other at p≤0.05.–indicates that the corresponding weed species was not recorded.

### Allometric and yield-related traits of maize crop

Maize crop recorded the highest values of LAI, CGR and root length at 35, 55, 75 and 95 DAS with PLM, while the lowest was recorded for WC treatment (Figs 3 and 4).

**Fig 3:** Impact of different mulching treatments on leaf area index and crop growth rate of maize crop. In the legend, WC = Weedy check (control), WF = Weed free (control), Pl-M = Plastic mulch, SM = Sorghum mulch, PM = Paper mulch.

**Fig 4:** Impact of different mulching treatments on root length of maize crop. In the legend, WC = Weedy check (control), WF = Weed free (control), Pl-M = Plastic mulch, SM = Sorghum mulch, PM = Paper mulch.

Sunflower crop had the highest values of LAI, CGR and root length with PLM at all data sampling dates as compared to the lowest values in WC treatment (Figs 5 and 6). Periodic data indicated that LAI and CGR of both crops improved from 35–55 DAS and then started to decline (Figs 3 and 5).

**Fig 5:** Impact of different mulching treatments on leaf area index and crop growth rate of sunflower crop. In the legend, WC = Weedy check (control), WF = Weed free (control), Pl-M = Plastic mulch, SM = Sorghum mulch, PM = Paper mulch.

**Fig 6:** Impact of different mulching treatments on root length of sunflower crop. In the legend, WC = Weedy check (control), WF = Weed free (control), Pl-M = Plastic mulch, SM = Sorghum mulch, PM = Paper mulch.

Different mulching treatments had significant effect on all yield-related traits of maize crop. All mulching treatments significantly influenced plant height of maize. The longest plants were noted for PLM and PM, while WC treatment resulted in the shortest plants (Table 3). The highest cob length was noted for PLM, which was statistically similar with PM, while WC treatment resulted in the lowest cob length (Table 3). The highest and the lowest number of grains per cob were recorded for PLM and WC treatments, respectively (Table 3). All mulch treatments had significant effect on 1000-grains weight of maize. The highest and the lowest 1000-grains weight was recorded for PLM and PM, and WC treatments, respectively (Table 3). The highest values of biological and grain yields were recorded for PLM against the lowest values for WC treatment (Table 3).

**Table 3:** Impact of different mulching treatments on yield-related traits of maize.

Treatments	Plant height (cm)	Cob length (cm)	Grains per cob	1000-grains weight (g)	Biological yield (t ha^-1^)	Grain yield (t ha^-1^)	Harvest index (%)
**Weedy-check**	176.52 c	12.73 c	270.67 c	290.33 c	12.74 d	5.50 e	44.15 b
**Weeds-free**	186.27 b	13.30 bc	324.67 b	301.67 b	14.30 c	7.09 d	47.40 a
**Plastic mulch**	210.33 a	15.60 a	403.67 a	318.33 a	16.93 a	9.61 a	47.06 a
**Sorghum mulch**	188.32 b	13.93 bc	346.33 b	303.67 b	14.76 c	7.78 c	42.87 b
**Paper mulch**	206.20 a	14.40 ab	360.00 b	311.33 a	15.90 b	8.43 b	44.69 ab
**LSD at p≤0.05**	7.38	4.92	5.78	7.03	2.72	3.21	2.72

Means not having common letter for individual and interactive effects significantly vary from each other at p≤0.05.

### Allometric and yield-related traits of sunflower crop

Different mulch treatments significantly influenced yield-related traits of sunflower. The longest plant height was noted for PLM and PM, while WC treatment observed the lowest plant height (Table 4). Mulch treatments positively influenced head diameter and achenes per head of sunflower. The highest values of head diameter and achenes per head were noted with PLM, whereas the lowest were recorded in WC treatment (Table 4). The highest 1000-achene weight was noted for PLM and PM which was statistically similar with SM, while WC recorded the lowest 1000-achene weight (Table 4). The highest biological and achene yields were recorded for PLM, whereas the lowest were noted in WC treatment (Table 4).

**Table 4:** Impact of different mulching treatments on yield-related traits of sunflower.

Treatments	Plant height (cm)	Head dimeter (cm)	Achenes per head	1000-achenes weight (g)	Biological yield (t ha^-1^)	Achene yield (t ha^-1^)	Harvest index (%)
**Weedy-check**	163.83 c	11.93 d	725.00 d	37.43 c	8.70 d	3.27 d	42.75 bc
**Weeds-free**	170.71 b	12.60 cd	764.67 c	46.44 b	10.67 c	4.08 c	41.35 c
**Plastic mulch**	185.50 a	15.07 a	915.33 a	53.26 a	14.57 a	6.75 a	45.53 ab
**Sorghum mulch**	168.40 bc	13.03 bc	789.67 c	49.46 ab	12.01 bc	5.39 b	45.74 ab
**Paper mulch**	180.90 a	13.83 b	841.33 b	51.20 a	12.58 b	5.80 b	46.13 a
**LSD at p≤0.05**	5.33	3.87	1.67	5.10	2.72	6.461	3.90

Means not having common letter for individual and interactive effects significantly vary from each other at p≤0.05.

## Discussion

Different mulch treatments used in the study significantly influenced weeds’ diversity, and density of total, broadleaved, grassy, and individual weed species in both crops (Fig 2, Tables 1 and 2). However, our hypothesis that SM will provide better control over weed flora compared to other mulching treatments was not supported by the results. The reason for better suppression of weed flora by PLM is the color of the plastic which did not allow light penetration; hence, seed germination of weeds was retarded. Furthermore, solarizing effect of the PLM probably increased temperature and decreased the viability of weed seeds. However, no such data is available to support this claim. Different mulches used to control the emergence of weed species act as physical obstacles [46], for essential resources like oxygen, light, nutrients, and water. The similar actions were performed by the mulches used in the current study. However, PLM proved better as lesser light penetration and conserved soil moisture both resulted in lower weed infestation and high productivity of both crops, respectively. Moreover, irrigation water negatively influenced SM (opened places for light penetration and weed emergence) and PM (the paper gets dissolved with time), while PLM remained unaffected. Significant control over weed through the use of mulches has been reported in an earlier studies [39–41,47]. The PLM performed better for suppressing weed flora (Tables 1 and 2). It might be linked with its longer life and less permeability compared to the rest of the mulch materials included in the current study. Narayan et al. [48], reported that density of weeds was significantly reduced and moisture retention improved by black plastic mulch as compared to other colors of plastic mulches.

Mulching treatments significantly improved allometric traits, i.e., LAI and CGR of maize and sunflower (Figs 3 and 5). It can be linked with better weed control and water conservation provided by the mulch treatments. Plastic mulches can effectively improve crop growth by controlling weeds, modified soil temperature and moisture [28,48]. Plant morphology and physiological metabolism significantly influenced by light intensity, spectral energy, light quality, and photoperiod [49]. The photosynthetic activity of crops has been reported to increase by using suitable-colored mulches, which improve dry matter accumulation and yield [50]. Therefore, PLM improved LAI and CGR in this study owing to improved photosynthesis.

Mulching treatments, especially PLM, significantly improved root length of both crops (Figs 4 and 6). Root length is an important parameter associated with immersion of nutrients and moisture as roots are directly correlated with the growth of above-ground parts and grain yield [51]. It has been reported by several studies that soil temperature and moisture can be improved by using different types of mulches, i.e., PLM or SM [52], which improves stand establishment and crop development [53,54] and yield [55] as soil structure [56] and weed infestation [30] is suppressed by mulching.

Different mulching treatments, especially PLM improved yield and related traits of maize and sunflower. It may be due to lower weed infestation and moisture conservation provided by PLM. The PLM improves photosynthetic rate and CO_2_ assimilation, which are positively correlated with better LAI, photosynthetically active radiation, temperature, soil water content and root water transport [54]. The LAI indicates the size of assimilatory system of any crop and higher LAI is recorded for the plants which utilized more solar radiation for C assimilation. Higher LAI provides additional area for photo-assimilation ensuing more CGR. This higher assimilatory system because of more LAI and CGR give rise to more dry matter yield, and plant height, number of grains per cob, achenes per head and 1000-grain/achenes weight which finally enhanced yield of maize and sunflower. Similar results were also reported by Hu et al. [57], that ridge-sown crop yield was significantly improved by using plastic film mulch.

## Conclusion

The results revealed that different mulch materials significantly differed in their ability to suppress weed flora and improve the productivity of maize and sunflower. Plastic mulching resulted in the highest suppression of weed flora. Moreover, better allometric and yield-related traits of both crops were noted with plastic mulch. Therefore, it is recommended to use plastic mulch for suppressing weed flora and improving yield of maize and sunflower crops.

## Supporting information

S1 Table Minimal dataset of the study used to analyze, report, and interpret the results. (XLSX)
